This article has been retracted.

# MicroRNA-92b inhibits epithelial-mesenchymal transition-induced migration and invasion by targeting Smad3 in nasopharyngeal cancer

**DOI:** 10.18632/oncotarget.21342

**Published:** 2017-09-27

**Authors:** Chong Zhao, Feipeng Zhao, Huajun Feng, Shengen Xu, Gang Qin

**Affiliations:** ^1^ Department of Otolaryngology Head and Neck Surgery, The Affiliated Hospital of Southwest Medical University, Luzhou, Sichuan, P.R. China

**Keywords:** microRNA-92b, nasopharyngeal carcinoma, Smad3, EMT, invasion

## Abstract

Increasing studies reports that aberrant miRNAs contribute to nasopharyngeal carcinoma (NPC) development and progression. However, the role of miR-92b in NPC remains unclear. In present research, we found that a reduced miR-92b expression in NPC tissues and cell lines. The clinical data showed that the down-regulated miR-92b expression was obviously associated with adverse prognostic characteristic. Furthermore, we confirmed that miR-92b was a novel independent prognostic symbol for predicting 5-year survival of NPC patients. MiR-92b overexpression inhibited cell migration, invasion and EMT progress, while down-regulated miR-92b reversed the effect. Besides, miR-92b could modulate Smad3 by directly binding to its 3’-UTR. In clinical samples of NPC, miR-92b inversely correlated with Smad3. Alternation of Smad3 expression at least partially abrogated the migration, invasion and EMT progress of miR-92b on NPC cells. In summary, our results indicated that miR-92b functioned as a tumor suppressor gene in regulating the EMT and metastasis of NPC via targeting Smad3, and may represent a novel potential therapeutic target and prognostic marker for NPC.

## INTRODUCTION

Nasopharyngeal carcinoma (NPC) is a common highly malignant head and neck cancer derived from the epithelium of nasopharynx. It is prevalent in southern China and Southeast Asia [1, 2]. Although technical improvements in diagnostic technology and clinical treatment, including radiotherapy and chemotherapy, the long-term survival prognosis of NPC is still poor due to the local recurrence and early metastasis [3, 4]. Thus, it is critical to elucidate the underlying mechanisms of tumorigenesis and invasiveness and identify novel therapeutic marker and develop new efficient treatment.

MicroRNAs (miRNAs) are a family of single-stranded and non-coding small RNAs with sequence lengths of 19-25 nucleotides. MiRNAs regulate the translation and degradation of target mRNA by binding with complementary sequences within the 3’-untranslated region (UTR) [5-7]. Recently, accumulating studies have reported that abnormal miRNAs are involved in several biological processes [8], including proliferation, apoptosis, and metastasis, and could serve as therapeutic response and prognostic biomarkers for NPC.

Recent evidence demonstrated that miR-92b was dysregulated in cancers [9, 10]. Huang et al reported that miR-92b targets DAB2IP to promote epithelial-mesenchymal transition (EMT) in bladder cancer migration and invasion [11]. MiR-92b promoted tumor proliferation, migration and invasion by targeting RECK in osteosarcoma [12, 13]. MiR-92b promotes tumor growth and activation of NF-ΚB signaling via regulation of NLK in oral squamous cell carcinoma [14]. Moreover, miR-92b promotes hepatocellular carcinoma progression by targeting Smad7 and is mediated by long non-coding RNA XIST [15]. These studies revealed that miR-92b play an oncogene in cancers. However, miR-92b was down-regulated in esophageal squamous cell carcinoma by targeting RAB23 [16]. MiR-92b was decreased and inhibited metastasis of non-small cell lung cancer by regulating Twist [17]. Thus, the functional significance of miR-92b in cancer initiation, development and process seems to be cancer-type specific. However, the functional effects and the underlying molecular mechanism by which miR-92b regulates the development and progression of NPC have not been elucidated.

Epithelial-to-mesenchymal transition (EMT), which was character of converting epithelial cells into mesenchymal cells, plays an important role in the biological progression for invasiveness and metastasis of cancers, including NPC. The typical EMT process usually decreases the cell adhesion molecule E-cadherin, which is an important determinant of epithelial cell-cell adhesion, while increases the Vimentin and N-cadherin expression, which are the mesenchymal markers. However, the relationship between miR-92b and EMT in NPC is poorly investigated.

In present study, we tried to explore the biological function of miR-92b in NPC progression. We demonstrated that miR-92b was decreased in both NPC tissues and cell lines. The down-regulated miR-92b was associated with adverse prognostic characters and poor 5-year survival of NPC patients. MiR-92b inhibited NPC migration and invasion *in vitro* by gain- and loss-of-function experiments through directly targeting Smad3. Moreover, our data revealed that miR-92b could suppressed EMT in NPC. In conclusion, these results elucidate the underlying mechanism by which miR-92b inhibits migration and invasion of NPC and propose miR-92b as a novel prognostic biomarker for NPC patients.

## RESULTS

### miR-92b is down-regulated in NPC tissues and cell lines

To determine the expression of miR-92b in NPC, we performed qRT-PCR to confirm that miR-92b expression was down-regulated in NPC tissues compared to normal nasopharyngeal epithelial tissues (P<0.05, Figure 1A). Furthermore, the expression of miR-92b was significantly decreased in a group of NPC cell lines (6-10B, CNE1, CNE2 and 5-8F) as compared with normal nasopharyngeal epithelial cell line NP69 (P<0.05, Figure 1B). Taken together, these data suggest miR-92b was down-regulated in NPC.

**Figure 1:** miR-92b is down-regulated in NPC Comparing differences in the expressions of miR-92b between **(A)** NPC and matched tumor-adjacent tissues and **(B)** NPC cell lines and the immortalized normal NP69. ^*^P < 0.05, ^**^P < 0.01.

### Clinical outcome of miR-92b expression in NPC patients

To explore the importance of miR-92b in the clinical features and prognosis of NPC patients, we measured miR-92b expression in eighty-nine samples using qRT-PCR and determined the different miR-92b expression according to the median value. As shown in Table 1, the reduced miR-92b was significantly associated with advanced T status (P = 0.008), distant metastasis (P = 0.023) and increased clinical stage (P = 0.004) (Table 1). Furthermore, in NPC patients, Kaplan-Meier survival analysis showed that high miR-92b expression was obviously correlated with better overall survival (OS) (P<0.01, Figure 2A) and disease-free survival (DFS) (P<0.01, Figure 2B). In addition, miR-92b was an independent prognostic factor for predicting 5-year OS and DFS in NPC patients (P=0.027, 0.022, respectively, Table 2). Taken together, these data indicate that down-regulated miR-92b expression is associated with disease progression in NPC.

**Table 1:** Comparison between the clinicopathological features and miR-92b expression in NPC (n = 89)

Clinical parameters	Cases (n)	Expression level		P value (^*^ p<0.05)
		miR-92b^high^(n=44)	miR-92b^high^(n=45)	
Age (years)				
< 50 years	49	23	26	0.602
≥50 years	40	21	19	
Gender				
Male	67	34	33	0.667
Female	22	10	12	
Histologic type				0.714
NKC	8	3	5	
KSCC	81	41	40	
T stage				0.008^*^
T1-2	48	30	18	
T3-4	41	14	27	
Clinical stage				0.004^*^
I+II	49	31	18	
III+IV	40	13	27	
Lymph metastasis				0.023^*^
positive	19	5	14	
negative	70	39	31	

KSCC, keratinizing squamous cell carcinoma; NKC, non-keratinizing carcinoma; NPC, nasopharyngeal carcinoma.

**Figure 2:** The prognostic value of miR-92b for NPC patients NPC patients with lower expression of miR-92b had worse **(A)** overall survival and **(B)** disease-free survival. The different miR-92b expression group was defined according to the median value 0.14. ^**^P<0.01.

**Table 2:** Significant prognostic factors by multivariate Cox regression analysis of 5-year overall and disease-free survival

Variables	Overall survival			Disease-free survival		
	HR	95% CI	*P*	HR	95% CI	*P*
miR-92b	0.357	0.105-0.948	0.027^*^	0.451	0.147-0.975	0.022^*^
T stage	2.341	1.128-5.652	0.011^*^	2.215	1.138-4.674	0.014^*^
Clinical stage	3.345	2.241-5.974	0.005^*^	3.482	2.244-6.346	0.004^*^
Lymph metastasis	3.576	1.254-6.211	0.017^*^	1.892	1.266-7.865	0.016^*^

HR, hazard ratio; CI, confidence interval; ^*^ statistically significant.

### miR-92b inhibits NPC migration and invasion *in vitro*

To investigate the effects of miR-92b on cell migration and invasion, we performed gain and loss-of-function experiment in 5-8F and CNE1 cells which contained the lowest and highest endogenous miR-92b. As measured by qRT-PCR, the transfection efficiencies were verified by knockdown and overexpression assays (P<0.05, Figure 3A and 3C). Firstly, we evaluated cell growth by MTT assays and found no significant difference after altering miR-92b expression in NPC cells (Supplementary Figure 1). We performed transwell migration and invasion assays to confirm that miR-92b overexpression significantly inhibited the migration and invasion of 5-8F cells (P<0.05, respectively, Figure 3B), while miR-92b knockdown markedly increased the number of migrated and invaded CNE1 cells (P<0.05, respectively, Figure 3D). These results emphasize the vital role of miR-92b in NPC cell migration and invasion.

**Figure 3:** miR-92b inhibits NPC cell migration and invasion *in vitro* **(A)** 5-8F cells that were transfected with corresponding miRNA vectors were subjected to qRT-PCR for miR-92b. **(B)** Cell migration and invasion as measured by Transwell assays were inhibited by overexpression of miR-92b in 5-8F cells. **(C)** CNE1 cells that were transfected with miR-92b inhibitors (anti-miR-92b) and negative control were subjected to qRT-PCR for miR-92b. **(D)** Cell migration and invasion as measured by Transwell assays were increased by knockdown of miR-92b in CNE1 cells. n = six independent experiments. ^*^P<0.05, ^**^P<0.01.

### miR-92b suppresses NPC epithelial-to-mesenchymal transition phenotype

Epithelial-mesenchymal transition (EMT) plays an important role in the metastasis process of NPC. To indicate the potential role of miR-92b in EMT process, western blot was performed and the data showed that miR-92b overexpression promoted epithelial marker E-cadherin and inhibited the mesenchymal marker N-cadherin and Vimentin expression in 5-8F cells (P<0.05, Figure 4A). In contrary, miR-92b knockdown decreased E-cadherin and increased N-cadherin and Vimentin expression in CNE1 cells (P<0.05, Figure 4B). Moreover, we explored the relationship between miR-92b and E-cadherin, Vimentin in NPC tissues, we performed IHC to confirm that the E-cadherin expression in miR-92b high expressing NPC tissues was higher than that in low miR-92b expressing tissues. Nevertheless, Vimentin expression in high miR-92b group was significantly lower than that in low miR-92b group (P<0.05, Figure 4C). In conclusion, these data indicated that miR-92b regulates EMT process in NPC.

**Figure 4:** miR-92b suppresses epithelial-to-mesenchymal transition in NPC cell The overexpression of miR-92b in 5-8F cells increased the expression of the epithelial cell marker E-cadherin and decreased the expression of the mesenchymal cell marker N-cadherin and Vimentin **(A)**. In contrast, the expression of the antagomiR to miR-92b decreased E-cadherin expression and increased N-cadherin and Vimentin expression **(B)**. **(C)** Immunohistochemical analysis of E-cadherin and Vimentin in NPC samples. In cases of high miR-92b expression; there was strong E-cadherin (left, up) and no detectable Vimentin protein (left, down) expression in the same tissue section. In contrast, in the case of low miR-92b expression, there was no detectable E-cadherin (right, up) and strong Vimentin protein (right, down) expression. Values are depicted as mean ± SEM; ^*^P < 0.05 by t test.

### Smad3 is a direct target of miR-92b in NPC cells

We used bioinformatic analysis (TargetScan and miRanda) to search the potential target of miR-92b and found Smad3 contained the putative binding site for miR-92b in its 3’-UTR (Figure 5A). To determine whether Smad3 is a target of miR-92b, we performed luciferase assays and confirmed that miR-92b overexpression significantly decreased the luciferase activity of wild-type (wt) Smad3 3’-UTR (P<0.05, Figure 5B) while had no influence on that of mutant (mt) Smad3 3’-UTR. In contrary, miR-92b knockdown increased the luciferase activity of wt Smad3 3’-UTR (P<0.05, Figure 5B) but did not affect the luciferase activity of mt Smad3 3’-UTR constructs. Moreover, we performed qRT-PCR and Western blot assays to check that miR-92b overexpression significantly inhibited, while miR-92b knockdown promoted the mRNA and protein of Smad3 in NPC cells (P<0.05, respectively, Figure 5C and 5D). These results indicated that Smad3 is a direct target of miR-92b.

**Figure 5:** Smad3 is identified as a direct target of miR-92b in NPC **(A)** miR-92b and its putative binding sequence in the 3’-UTR of Smad3. The mutant binding site was generated in the complementary site for the seed region of miR-92b. **(B)** miR-92b significantly suppresses the luciferase activity that carried wild-type (wt) but not mutant (mt) 3’-UTR of Smad3. Anti-miR-92b led to a notable increase in the luciferase activity of wt 3’-UTR of Smad3. **(C)** qRT-PCR analysis of Smad3 mRNA expression in 5-8F cells with miR-92b or miR-control vector transfection and CNE1 cells with anti-miR-92b or anti-miR-NC vector transfection. **(D)** Overexpression of miR-92b reduced the expression of Smad3 protein in 5-8F cells and knockdown of miR-92b increases the level of Smad3 protein in CNE1 cells. n = six repeats with similar results, ^*^P<0.05, n.s: no significance.

### miR-92b inversely correlated with Smad3 expression in NPC tissues

To further explore the relationship between miR-92b and Smad3 in NPC tissues, we measured the Smad3 mRNA and protein expression in different expression levels of miR-92b. Our data revealed that both Smad3 mRNA and protein expression level in high miR-92b group were significantly lower than that in low miR-92b group in NPC (P<0.05, Figure 6A and 6B). Moreover, we demonstrated that the mRNA level of Smad3 in the NPC tissues was inversely correlated with miR-92b expression (R^2^=0.6548, P<0.0001, Figure 6C). Similarly, as measured by IHC assay, Smad3 protein expression in miR-92b high-expressing tumors was obviously lower than miR-92b low-expressing tumors (P<0.05, Figure 6D). In addition, we performed western blot and confirmed the expression of Smad3 in NPC tissues was significantly higher than that in non-tumor tissues (P<0.05, Supplementary Figure 2). Taken together, these data suggest that Smad3 was a direct downstream of miR-92b in NPC.

**Figure 6:** An inverse correlation between miR-92b and Smad3 expression is observed in NPC **(A)** The expression of Smad3 mRNA in miR-92b high-expressing tumors was significantly lower than that in miR-92b low-expressing tumors. **(B)** The expression of Smad3 protein in miR-92b high-expressing tumors was significantly lower than that in miR-92b low-expressing tumors. **(C)** A significant inverse correlation between the mRNA levels of Smad3 and miR-92b was observed in NPC tissues. **(D)** Representative immunohistochemical staining showed a weak staining of Smad3 in miR-92b high-expressing NPC tissue and strong staining of Smad3 in the miR-92b low-expressing tumor. ^*^P<0.05.

### Inhibition of Smad3 mimics miR-92b-induced migration and invasion

After confirming that Smad3 is a target of miR-92b, we next explore the biological function of Smad3 in NPC, we transfected NPC cell line CNE1 with empty vector (EV) or Smad3 plasmids (P<0.01. Figure 7A). We demonstrated that Smad3 overexpression prominently promoted NPC cell migration and invasion in CNE1 (P<0.05. Figure 7B). Moreover, Smad3 was knocked down using a specific siRNA in 5-8F cells (P<0.05. Figure 7C). As expected, down-regulated Smad3 led to a significant reduction of cell migration and invasion (P<0.05. Figure 7D). These data suggest that Smad3 regulates the migration and invasion of NPC cells and inhibition of Smad3 expression could mimic the effect of miR-92b.

**Figure 7:** Smad3 promotes NPC cell migration and invasion **(A)** CNE1 cells that were transfected with empty vector **(EV)** or Smad3 plasmids were subjected to western blot for Smad3. n = six independent experiments; ^*^P < 0.05 by t test. **(B)** Cell migration and invasion as measured by Transwell assays were increased by Smad3 overexpression in CNE1 cells as compared with control cells. n = three repeats with similar results, ^*^P < 0.05 by t test. HPF: high power field. **(C)** 5-8F cells that were transfected with scrambled siRNA or Smad3 siRNA were subjected to western blot for Smad3. n = six independent experiments; ^*^P < 0.05 by t test. **(D)** Smad3 knockdown 5-8F cells conferred a less number of migrated and invaded cells as compared with control cells. n = three repeats with similar results; ^*^P < 0.05 by t test. HPF: high power field.

### Altering Smad3 expression reverses the biological function of miR-92b on NPC cell migration, invasion and EMT process

To explore that Smad3 is a functional mediator of miR-92b, we restored Smad3 by overexpression plasmids in miR-92b-overexpressing 5-8F cells (P<0.05, Figure 8A). Smad3 restoration abrogated the inhibitory effects of miR-92b on migration and invasion of 5-8F cells (P<0.05, respectively, Figure 8B). Similarly, Smad3 knockdown by a specific siRNA in miR-92b-suppressive CNE1 cells significantly reversed the promoting function induced by miR-92b loss on CNE1 cell migration and invasion (P<0.05, respectively, Figure 8C and 8D). Furthermore, altering Smad3 expression mediated the effects of miR-92b on EMT events in NPC cells (P<0.05, respectively, Figure 8E and 8F). These data demonstrated that Smad3 is not only a downstream target, but also a functional mediator of miR-92b in NPC.

**Figure 8:** Alterations of Smad3 partially abolish miR-92b-mediated NPC cell migration, invasion and EMT progress **(A)** miR-92b-overexpressing 5-8F cells that were transfected with EV or Smad3 expression plasmid were subjected to western blot analysis for Smad3. **(B)** Cell migration and invasion of the miR-92b-overexpressing 5-8F cells was increased by Smad3 overexpression. **(C)** miR-92b-suppressive CNE1 cells that were transfected with control siRNA or Smad3 siRNA were subjected to western blot analysis for Smad3. **(D)** Smad3 knockdown abrogated the effects of miR-92b knockdown on CNE1 cells. **(E)** Western blot analysis of EMT marker proteins in 5-8F cells stably expressing miR-92b transduced with Smad3 or control vector. **(F)** Western blot analysis of indicated proteins in CNE1 cells stably expressing miR-92b inhibitor transfected with Smad3 siRNA or control siRNA. n = six independent experiments. EV, empty vector. ^*^P<0.05.

## DISCUSSION

MiRNAs have been identified as tumor suppressors or oncogenes through modulation of target genes during cancer initiation and development [18], including NPC [19-21]. The miRNA expression was treated as approach for preparation of prognostic biomarkers and effective therapeutic targets of NPC [22, 23]. MiR-92b was recently identified as a novel cancer-related miRNA [24-26]. MiR-92b regulates the cell growth, cisplatin chemosensitivity of A549 non-small cell lung cancer and target PTEN [27]. In glioblastomas, miR-92b functions as a potential oncogene by targeting Smad3 [28]. MiR-92b inhibitor promoted glioma cell apoptosis via targeting DKK3 and blocking the Wnt/beta-catenin signaling pathway [29]. Moreover, miR-92b regulates glioma cells proliferation, migration, invasion and apoptosis via PTEN/AKT signaling pathway [30]. In present research, we found that miR-92b was significantly down-regulated in NPC tissues and cell lines. Reduced miR-92b expression was obviously correlated with malignant clinicopathological features of NPC patients, including advanced T status, distant metastasis and increased clinical stage. Moreover, survival analysis showed that high miR-92b group had a significant better 5-year OS and DFS for NPC patients. Multivariate Cox repression analysis indicated that miR-92b was an independent prognostic factor for predicting survival of NPC patients. These data indicate that miR-92b was identified as a promising biomarker for predicting prognosis of NPC patients.

Local recurrence and distant metastasis are the major cause of treatment failure and NPC related deaths [31]. In this study, miR-92b overexpression inhibited the migration and invasion of NPC cells while miR-92b knockdown increased these metastatic behaviors *in vitro* by gain- and loss-of-function experiment. EMT is a critical process in the metastasis of NPC [32]. We demonstrated that miR-92b suppressed EMT progress of NPC cells. These results suggest that miR-92b inhibits NPC metastasis by suppressing EMT phenotype.

In NPC, TGF-β/Smad signaling pathway play a crucial role in cancer metastasis. Smad3 is a modulator of TGF-β signaling [19, 33, 34]. We used prediction algorithms to Smad3 is a putative target of miR-92b. We confirmed that Smad3 was a direct downstream target of miR-92b and mediated the metastasis and EMT progress in NPC. Moreover, we confirmed that alteration of Smad3 could mimic the effects of miR-92b on migration and invasion of NPC. The restoration of Smad3 in NPC cells prominently reversed tumor migration, invasion and EMT mediated of miR-92b. Taken together, Smad3 is not only a downstream target but also a possible mediator of miR-92b in NPC.

In conclusion, we demonstrated that miR-92b was down-regulated in NPC tissues and cell lines, and its reduced expression was correlated with malignant clinicopathological features. Furthermore, we confirmed miR-92b inhibited cell migration, invasion and EMT by inhibiting Smad3. These results suggest that miR-92b is a potential metastasis-associated tumor suppressor in NPC. Collectively, the deregulation of miR-92b may play an important role in tumor metastasis and may be a novel prognostic factor and potential therapeutic target for NPC.

## MATERIALS AND METHODS

### NPC specimens and cell culture

89 NPC tissues and 20 normal nasopharyngeal tissues were obtained from Department of Otolaryngology Head and Neck Surgery, the Affiliated Hospital of Southwest Medical University during January 2011 to December 2016. All NPC patients did not receive perioperative radiotherapy or chemotherapy before surgery. Written informed consents were obtained from all patients enrolled in this study. The demographic and clinicopathologic features of all patients were shown in Table 1. The Ethics Committee of Southwest Medical University approved all protocols involving patients’ samples according to the Declaration of Helsinki (as revised in Tokyo 2004).

Human NPC cell lines 5-8F, 6-10B, CNE-1 and CNE-2 were cultured in RPMI-1640 (Gibco, Grand Island, NY, USA) containing 10% fetal bovine serum (Gibco, USA), 100 U/mL penicillin, and 100 U/mL streptomycin. The human immortalized nasopharyngeal epithelial cell line NP69 were cultured in serum-free medium (Invitrogen) supplemented with all necessary growth factors (Gibco, USA). All cells were maintained in a humidified cell incubator with 5% CO2.

### Real-time quantitative PCR

Trizol (Invitrogen) was used to extract the RNA from clinical specimens and NPC cells following the manufacturer’s instruction. PCR amplification and quantification for miR-92b was performed using the TaqMan miRNA Reverse Transcription Kit (Applied Biosystms, Foster City, CA, USA) and TaqMan Human MiRNA Assay Kit (Applied Biosystems, Foster City, CA, USA). Primers against miRNA miR-92b (HmiRQP0835) and U6 (HmiRQP9001) were purchased from Genecopoeia (Guangzhou, China). U6 was used as the internal control for measuring the relative level of miR-92b.

### Western blot

Cellular proteins extracted from NPC cells using RIPA lysis buffer (BioMed, China) were separated in SDS-PAGE gels and were transferred to PVDF membrane. The blots were incubated with the following primary antibodies overnight: GAPDH (1:2,500, Cell Signaling Technologies, Danvers, MA, USA), and Smad3 (1:500, Santa Cruz). After incubating with the primary antibody, the membranes were incubated with secondary antibodies (1: 5,000; Bio-Rad, USA) at room temperature for 2 hours, then the protein signal were detected using the Bio-Rad Gel imaging system.

### Transwell assays

1 × 10^5^ NPC cells transfected with corresponding vectors were re-suspended in serum-free medium and were seeded into the transwell inserts of 8-μm with (Millipore, USA). 650 ul Serum-containing medium (20% FBS) was used in the lower chamber as the attractant. Regarding the invasion assay, each upper chamber was coated with mixture of DMEM and Matrigel (Becton Dickinson Labware, USA) at a ratio of 8:1. 24 hours later, the NPC cells migrated or invaded through the transwell membranes were on the lower surface and were stained with 0.1% crystal violet, and the cell numbers were obtained from 10 different fields of the lower surface of the filter. Three independent experiments were performed.

### Luciferase reporter assay

Wild-type Smad3 3’-UTR sequence and the mutated Smad3 3’-UTR sequence were constructed into the pGL3 control vector (Promega, USA) to get wt Smad3-3’-UTR vector and mt Smad3-3’-UTR vector, respectively. For luciferase reporter assay, NPC cells were co-transfected with the wild type construct or mutant construct, and, miR-92b mimics or inhibitor or control or negative control vector. 48 hours after transfection, cells were harvested and lysed. The Dual-Luciferase Reporter Assay system (Promega, Shanghai, China) were used to the firefly and Renilla luciferase activities.

### Cell transfection

MiRNA vectors, including precursor miR-92b clones (HmiR0015), precursor miR-92b scrambled control clones (miR-control; CmiR0001), miR-92b inhibitors (anti-miR-92b; HmiR-AN0835) and miR-92b inhibitor control clones (anti-miR-NC; CmiR-AN0001) were obtained from Genecopoeia (Guangzhou, China). The Smad3 overexpression plasmid and specific siRNA against Smad3 and a control siRNA were synthesized by Sangon Biotech Co., Ltd. (Shanghai, China). Cells were transfected with above vectors using Lipofectamine 2000 Reagent (Invitrogen Life Technologies) in accordance with the manufacturer’s protocol.

### Immunohistochemistry (IHC)

Briefly, 4 μm sections were deparaffinized in xylene, rehydrated through graded ethanols, followed by blocking of endogenous peroxidase activity in 3% hydrogen peroxide for 10 min at room temperature. The corresponding antibody (1:300, Cell Signaling Technology, Inc.) was applied as the primary antibody by a streptavidin peroxidase-conjugated (SP-IHC) method. The staining results were semi-quantitatively evaluated by the multiply of staining intensity and the percentage of positive staining cells. The percentage of positive cells was given into four grades: 0 for <5%; 1 for 6%–25%; 2 for 26%–50%; 3 for 51%–75% and 4 for >75%. Staining intensity was assessed by four degrees: 0, negative; 1, weak; 2, moderate; and 3, strong. Each section was assayed for ten independent high magnifications (×400) fields to get the average scores.

### Statistical analysis

Data are presented as the mean ± SD and performed at least three independent replicates. SPSS software, 16.0 (SPSS, Inc, Chicago, IL, USA) and Graphpad Prism 6.0 (CA, USA) were used for a two-tailed Student t-test, Pearson’s correlation analysis, Kaplan-Meier method and the log-rank test to evaluate the statistical significance. Differences were defined as P<0.05.

## SUPPLEMENTARY MATERIALS FIGURES


